This article has been retracted.

# Effect of Cryotherapy plus Flurbiprofen Axetil for Pain Management in Children Undergoing Tonsillectomy

**DOI:** 10.1155/2022/7687437

**Published:** 2022-07-14

**Authors:** Ping Gao, Wenyun Wang, Wenhui Yang, Tingting Yan, Biaoxin Zhang

**Affiliations:** ^1^School of Nursing, Anhui Medical University, Department of Emergency Medical, The First Affiliated Hospital of USTC, Division of Life Sciences and Medicine, University of Science and Technology of China, Hefei 230032, China; ^2^Department of Anesthesiology, The First Affiliated Hospital of USTC, Division of Life Sciences and Medicine, University of Science and Technology of China, Hefei 230001, China; ^3^Department of Otolaryngology Head and Neck Surgery, The First Affiliated Hospital of Anhui Medical University, Hefei 230032, China

## Abstract

**Objective:**

To investigate the effect of cryotherapy using ice pops for physical analgesia and preventive analgesia using flurbiprofen axetil for pain management in children undergoing tonsillectomy.

**Methods:**

A total of 120 children scheduled for tonsillectomy were recruited after assessment for eligibility and assigned to a control group (group *C*), flurbiprofen axetil group (group *F*), cryotherapy group (group *I*), and cryotherapy plus flurbiprofen axetil group (Group FI) via the random number table method. Groups *F* and FI were given 1 mg/kg of flurbiprofen axetil through intravenous injection 30 min before surgery, while group *C* received an equal amount of saline at the same time point. Groups *I* and FI received sweet ice pops for pain relief after recovery from anesthesia. The modified Children's Hospital of Eastern Ontario Pain Scale (mCHEOPS) scores and pediatric anesthesia emergence delirium (PAED) scores at 5 minutes (T1), 30 minutes (T2), 60 minutes (T3), 4 hours (T4), and 24 hours (T5) postoperatively, and the incidence of postoperative complications in the children were recorded by investigators who were masked to the grouping results.

**Results:**

From T1 to T4, significantly lower mCHEOPS scores and PAED scores were observed in group F, group *I*, and group FI versus those in group *C* (*P* < 0.05). At T2, group FI showed significantly lower mCHEOPS scores and PAED scores versus groups F and I (*P* < 0.05). There were no significant differences in the mCHEOPS scores and PAED scores between the four groups at 24 h postoperatively (*P* > 0.05). The differences in the documented postoperative complications between the four groups did not come up to the statistical standard (*P* > 0.05).

**Conclusion:**

Cryotherapy plus flurbiprofen axetil for pain management significantly mitigates post-tonsillectomy pain and delirium in children and facilitates recovery, with no significant adverse events.

## 1. Introduction

Tonsillectomy is a widely performed surgical procedure worldwide and is the second most common surgery performed on children [1]. Removal of the tonsils is possible in cases of recurrent acute tonsillitis, peritonsillar abscesses, and in young children, where the tonsils have become enlarged and hypertrophied, resulting in poor circulation of the upper respiratory tract and even difficulty in breathing and swallowing [2]. Other conditions, such as tonsillar keratosis and tonsillar tumours, can also be treated by this procedure [3]. Pain, bleeding, agitation, and dysphagia after tonsillectomy are the main factors affecting postoperative recovery [4]. The pain, mainly at the throat and the ears, builds up for the first few days and is usually at its worst around the fifth day after surgery. Intense pain is one of the most important postoperative complaints after tonsillectomy, and inadequate postoperative pain management is associated with negative consequences such as the development of chronic postoperative pain, impaired throat function, and negative psychological states.

Currently, pain management after tonsillectomy consists of physical analgesics, such as ice packs, and pharmacological management. Nonsteroidal anti-inflammatory drugs (NSAIDs) are privileged for pharmacological analgesia [5], and other drugs include preoperative dexmedetomidine nasal drip or local anesthetic application [6, 7]. Flurbiprofen ester reduces prostaglandin synthesis by inhibiting cyclooxygenase (COX) in the spinal cord and periphery, reducing the nociceptive hypersensitivity state caused by surgical trauma [8]. Lipid microsphere formulations are more potent, have a more rapid onset of action, last longer, and are less likely to cause adverse effects such as gastric mucosal damage [9]. Its use in postoperative analgesia has the advantage that it has no central depressant effect, does not interfere with the awakening of patients under anaesthesia, and can be used immediately after surgery [10]. However, relatively little knowledge is available related to the joint use of physical and pharmacological analgesia in children undergoing tonsillectomy. To this end, this study was undertaken to evaluate the clinical effects and safety of cryotherapy using ice pops for physical analgesia and preventive analgesia using flurbiprofen axetil for pain management in children undergoing tonsillectomy, so as to provide a reference for clinical application.

## 2. Materials and Methods

### 2.1. Baseline Patient Profile

120 children scheduled for tonsillectomy and/or adenoidectomy were recruited for prospective analysis and assigned by random number table to the control group (group *C*), flurbiprofen axetil group (group *F*), cryotherapy group (group *I*), and cryotherapy plus flurbiprofen axetil group (group FI). The experiments were approved by the ethics committee of The First Affiliated Hospital of USTC (no. FAHUSTC753). All participants' families were informed, and they signed the consent form.

Inclusion criteria were (1) patients aged 3–11 years; (2) patients with an American Society of Anesthesiologists (ASA) physical status classification of I-II [11] and normal cardiopulmonary, hepatic, and renal function; (3) no preoperative chronic pain.

Exclusion criteria were (1) history of NSAID drug allergy, recent peptic ulcer, neuromuscular sensory abnormalities, hepatic, renal, and haematological dysfunction; (2) patients who have used analgesics within the last 24 hours; (3) patients who have undergone another procedure for the above reasons.

### 2.2. Treatment Methods

The blood pressure, oxygen saturation, and electrocardiogram of the children were monitored before surgery. All children received 0.1 mg/kg of tropisetron intravenously before surgery. 1 mg/kg of flurbiprofen axetil was administered to groups FI and F 30 min before surgery, and an equal amount of saline was given to group *C* at the same time point. The general anesthesia was established using 0.05 mg/kg of midazolam, 0.4 ug/kg of sufentanil, 0.2 mg/kg of etomidate, and cisatracurium besylate. After tracheal intubation, the breathing machine was connected for respiratory control, and the tidal volume was maintained at 8–10 ml/kg. Combined intravenous-inhalation anesthesia was used for anesthesia maintenance, with continuous infusion of propofol and remifentanil, intermittent inhalation of 0.5% to 1% sevoflurane, and additional cisatracurium besylate as needed. The heart rate and blood pressure of the children were maintained within 30% of the preoperative baseline values, the anesthesia was terminated at the completion of the operation, and the children were immediately sent to the postanesthesia care unit (PACU). The tracheal tube was removed when the children could breathe freely and were hemodynamically stable, and the patients of the children were asked to accompany the children to PACU. Children in groups *I* and FI were given a sweet ice pop for physical analgesia for 5 minutes after extubation under the instruction of the medical staff. Children with postoperative modified Children's Hospital of Eastern Ontario Pain Scale (mCHEOPS) scores greater than 4 points were given flurbiprofen axetil at a dose of 1 mg/kg.

### 2.3. Outcome Measures

1. The operating time and volume of intraoperative bleeding in the children were recorded.
2. Postoperative pain in the children was assessed using mCHEOPS scores and postextubation agitation of the children was assessed using the pediatric anesthesia emergence delirium (PAED) scale [12]. Scoring criteria are shown in Tables 1 and 2. The mCHEOPS scores and PAED scores at 5 minutes (T1), 30 minutes (T2), 60 minutes (T3), 4 hours (T4), and 24 hours (T5) postoperatively were recorded by investigators who were blinded to the grouping results. The mCHEOPS scores consisted of 5 domains, each with a score of 0–10 points, and the score was proportional to the severity of pain. The PAED scores also consisted of 5 domains, each with a score of 0–20 points, and the score was proportional to the severity of agitation.
3. The occurrence of traumatic bleeding, nausea and vomiting, postoperative diarrhea, and fever was recorded 3 days after surgery. Traumatic bleeding was defined as bleeding that requires surgical intervention for hemostasis. Postoperative diarrhea was defined as the number of bowel movements ≥3 times/day with loose stools. A postoperative temperature >38.0°C was defined as a febrile case.

### 2.4. Statistical Analysis

All statistical analyses were performed with the use of SPSS 17.0. Normally distributed measurement data are expressed as the mean ± standard deviation; a *t*-test was used to determine the statistical significance of differences between the groups, and an ANOVA with repeated measure design was used for intragroup comparisons. Count data are expressed as the number of cases and percentages (%) and analyzed using the chi-square test. The rank-sum test was used for the comparison of rank data. Statistically significant results were defined as *P* < 0.05.

## 3. Results

### 3.1. Baseline Patient Characteristics and Intraoperative Indices

There were no significant differences in the baseline characteristics such as age, weight, and gender ratios, the operation time, and the intraoperative bleeding volume between the four groups of children (*P* > 0.05) (Table 3).

### 3.2. Postoperative Pain and Agitation

From T1 to T4, significantly lower mCHEOPS scores and PAED scores were observed in group *F*, group *I*, and group FI versus those in group *C* (*P* < 0.05). At T2, group FI showed significantly lower mCHEOPS scores and PAED scores versus groups F and I (*P* < 0.05) (Table 4).

### 3.3. Postoperative Complications

The differences in the occurrence of traumatic bleeding, nausea and vomiting, postoperative diarrhea, and fever between the four groups of children did not come up to the statistical standard (*P* > 0.05) (Table 5).

## 4. Discussion

Most children complain of severe pain after tonsillectomy, which compromises the quality of life and leads to reduced diet, dysphagia, dehydration, and possibly long-term behavioral and/or psychological alterations [13]. Postoperative pain also predisposes children to agitation during the recovery period, especially in the early stages of tracheal tube removal in the PACU. Therefore, the significance of the control of mitigation of postoperative pain in pediatric tonsillectomy has been established definitively.

The aim of this study was to evaluate the clinical effectiveness and safety of physical analgesia using ice lolly cryotherapy and prophylactic analgesia using flurbiprofen axetilin children undergoing tonsillectomy. Prophylactic analgesia refers to the reduction of postoperative pain by reducing the transmission of surgically induced pain stimuli to the centre and preventing central sensitisation by preemptive analgesic drugs. Flurbiprofen axetilis is a nonsteroidal anti-inflammatory drug that is commonly used clinically for prophylactic analgesia [14]. It can be used for postoperative pain relief in children, has a rapid onset of action, lasts for a long time, and has no significant side effects, which is relatively safe. The dosage of this drug should be strictly followed to avoid overdosing, which may affect the normal growth and development of the child [15]. In this study, children who received flurbiprofen axetilin combination with cryotherapy achieved the lowest pain scores and agitation scores, suggesting a synergistic effect of cryotherapy and prophylactic analgesia in post-tonsillectomy pain management.

There is considerable evidence to support the impact of cryotherapy on post-tonsillectomy pain management. Vieira et al. [16] reported that the use of 500 ml of saline at 5°C to 10°C for 3 and 6 days postoperatively reduced pain. Similar results were obtained by Shin et al. [17], who used 300 ml of saline at 5°C to relieve postoperative pain. The current data confirm that cryotherapy has a significant effect on pain relief and agitation in the early posttracheal extubation period. The mechanism of action of cryotherapy is that low temperatures reduce tissue congestion and swelling and lower the activation threshold of tissue damage receptors and the conduction rate of pain nerve signals [18]. In this study, children in Groups *I* and FI received sweet ice lollies, which would create localised hypothermia in the mouth and a sweet taste to soothe the child.

Flurbiprofen axetilis is a nonsteroidal anti-inflammatory drug with stable pharmacokinetics and no significant adverse complications when used in pediatric patients over 6 months of age [19], but it may impair platelet function and lead to increased surgical bleeding. Postoperative follow-up in this study showed that flurbiprofen axetil used 30 minutes before surgery as prophylactic analgesia did not increase trauma bleeding. Furthermore, the lack of difference in postoperative complications among the four groups of children also suggests that the combination of cryotherapy plus flurbiprofen axetil has a high safety profile.

However, at any time during treatment with all (NSAIDs), adverse reactions of gastrointestinal bleeding, ulceration, and perforation can occur, and the risk can be fatal [20]. When gastrointestinal bleeding or ulceration occurs in patients taking the drug, it should be discontinued. Clinical trials have shown that this product may cause an increased risk of serious cardiovascular thrombotic adverse events, myocardial infarction and stroke, the risk of which may also be fatal [21]. Patients with cardiovascular disease or risk factors for cardiovascular disease are at greater risk [22]. In Chinese medicine, the main ingredients of Du Liang soft capsules are Angelica dahurica and Rhizoma Chuanxiong, which is an orally administered proprietary Chinese medicine preparation [23]. The clinical effects are mainly to dispel wind and cold, invigorate blood, and promote blood circulation. The clinical effects are mainly for the treatment of headaches, and the TCM symptoms need to be of the type of wind-cold and blood stasis blocking the arteries and channels [24]. A study has demonstrated the efficacy of Du Liang soft capsule in relieving pain after hand tonsillectomy with no significant adverse effects, which provides another basis for the combined treatment of Chinese and Western medicine [25].

However, there are a number of limitations to this study. The number of popsicles consumed by children was not standardised, there were subjective judgements on postoperative pain and agitation scores, and the limited duration of postoperative follow-up did not allow for an objective evaluation of long-term outcomes. More scientific and precise indicators are needed for evaluation in follow-up trials.

## 5. Conclusion

Flurbiprofen axetil preventive analgesia is available for postoperative analgesia in children undergoing tonsillectomy, and ice pops offer an economical and safe alternative for short-term postoperative analgesia. Cryotherapy plus flurbiprofen axetil for pain management significantly mitigates post-tonsillectomy pain and delirium in children and facilitates recovery, with no significant adverse events.

## Figures and Tables

**Table 1:** Modified children's hospital of eastern Ontario pain scale scores.

Scores	0 points	1 point	2 points
Crying	None	Moaning	Screaming
Facial expressions	Smiling	Calm	Painful
Language	No pain	No complaint of pain	Complaint of pain
Body reaction	Normal	Relaxed	Nervous and quivering
Legs	Normal	Kicking	Need for constraints

**Table 2:** Pediatric anesthesia emergence delirium scores.

Items	4 points	3 points	2 points	1 point	0 points
Eye contact with their guardians	None	Infrequent	Moderate	Frequent	Extremelyfrequent
Behavioral purposefulness	None	Infrequent	Moderate	Frequent	Extremelyfrequent
Recognize the environment	None	Infrequent	Moderate	Frequent	Extremely frequent
Restlessness and agitation	Extremely frequent	Frequent	Moderate	Infrequent	None
Unmitigated crying	Extremely frequent	Frequent	Moderate	Infrequent	None

**Table 3:** Baseline characteristics and intraoperative indices ($\bar{x}\pm s$, *n* = 30).

Groups	*n*	Male/female	Age (year)	Height (cm)	Weight (kg)	Operation time (min)	Intraoperative bleeding volume (ml)
Group *C*	30	21/9	6.87 ± 2.73	121.28 ± 15.78	22.30 ± 8.15	78.37 ± 14.76	26.40 ± 8.17
Group *F*	30	19/11	6.70 ± 2.07	116.60 ± 11.78	23.28 ± 7.91	73.10 ± 16.43	23.37 ± 8.60
Group *I*	30	21/9	7.07 ± 2.38	116.42 ± 12.65	22.78 ± 8.64	76.45 ± 17.33	22.76 ± 6.76
Group FI	30	22/8	7.20 ± 2.57	120.00 ± 14.06	22.94 ± 8.89	75.53 ± 15.17	22.17 ± 7.03

**Table 4:** Postoperative pain and agitation ($\bar{x}\pm s$, *n* = 30).

Indices	Groups	*n*	*T*_1_	*T*_2_	*T*_3_	*T*_4_	*T*_5_
MCHEOPS scores	Group *C*	30	3.4 ± 0.8	3.4 ± 0.7	3.2 ± 0.7	2.2 ± 0.8	0.8 ± 0.4
	Group *F*	30	2.5 ± 0.6^a^	2.6 ± 0.8^a^	2.1 ± 0.9^a^	1.2 ± 0.5^a^	0.8 ± 0.5
	Group *I*	30	2.5 ± 0.7^a^	2.8 ± 0.9^a^	2.1 ± 0.8^a^	1.2 ± 0.5^a^	0.8 ± 0.4
	Group FI	30	2.2 ± 0.6^a^	1.8 ± 0.8^ab^	1.8 ± 0.8^a^	1.2 ± 0.4^a^	0.7 ± 0.5

PAED scores	Group *C*	30	6.7 ± 1.6	8.2 ± 2.4	7.8 ± 1.8	3.5 ± 1.8	1.5 ± 1.2
	Group *F*	30	5.8 ± 1.2^a^	6.3 ± 1.5^a^	6.2 ± 2.0^a^	2.4 ± 1.3^a^	1.6 ± 1.4
	Group *I*	30	5.4 ± 1.5^a^	5.2 ± 1.4^a^	6.4 ± 2.2^a^	2.6 ± 1.3^a^	1.2 ± 0.8
	Group FI	30	5.3 ± 1.6^a^	4.2 ± 1.3^ab^	6.4 ± 1.5^a^	2.2 ± 1.6^a^	1.2 ± 0.7

*Note*. ^a^ indicates a significant difference (*P* < 0.05) in comparison with group *C*; ^b^ indicates a significant difference (*P* < 0.05) in comparison with groups *F* and *I*.

**Table 5:** Postoperative complications (*n* [%], *n* = 30).

Groups	Traumatic bleeding	Nausea and vomiting	Postoperative diarrhea	Fever
Group *C*	2 (6.7)	2 (6.6)	0 (0)	3 (10.0)
Group *F*	1 (3.3)	1 (3.3)	1 (3.3)	4 (13.3)
Group *I*	0 (0)	2 (6.7)	0 (0)	2 (6.7)
Group FI	0 (0)	1 (3.3)	0 (8)	2 (6.7)

## Data Availability

No data were used to support this study.
